The article "The Effects of Letrozole and Metformin Combined with Targeted Nursing Care on Ovarian Function, LH, and FSH in Infertile Patients with Polycystic Ovary Syndrome" was published in 2022. Journal: J Healthc Eng.

# The Effects of Letrozole and Metformin Combined with Targeted Nursing Care on Ovarian Function, LH, and FSH in Infertile Patients with Polycystic Ovary Syndrome

**DOI:** 10.1155/2022/3712166

**Published:** 2022-03-23

**Authors:** Shuai Jiang, Ting Tang, Yongmei Sheng, Rui Li, Hua Xu

**Affiliations:** ^1^Reproductive Medicine Centre, Yantaishan Hospital, Yantai 264000, Shandong Province, China; ^2^Department of Emergency Medicine, Qingdao Eighth People's Hospital, Qingdao 266000, Shandong Province, China; ^3^Department of Emergency Medicine, Qingdao Hospital of Traditional Chinese Medicine, Hiser Medical Group of Qingdao, Qingdao 266033, Shandong Province, China; ^4^Department of Endocrinology, Zhangqiu Distrct People's Hospital, Jinan 250200, Shandong Province, China; ^5^Outpatient Operating Room, The Affiliated Qingdao Central Hospital of Qingdao University, The Second Affiliated Hospital of Medical College of Qingdao University, Qingdao 266042, Shandong Province, China

## Abstract

**Background:**

Polycystic ovary syndrome (PCOS) is a common gynecological endocrine disorder in women of gestational age and the most common cause of female infertility. This study aimed to investigate the effect of letrozole and metformin combined with targeted nursing on ovarian function, LH, and FSH in infertile patients with PCOS.

**Methods:**

A total of 72 infertile patients with PCOS were divided into the control group and combined group. The control group was given metformin tablets combined with targeted nursing therapy. The combined group was treated with letrozole on the basis of the control group. Ovarian function, LH, and FSH were compared between the two groups before and after treatment.

**Results:**

After treatment, the total effective rate (94.44%) of the combined group was significantly higher than that of the control group (80.56%). After treatment, the levels of HbA1c, FINS, HOMA-IR, TG, and TC in the two groups were lower than those before treatment, and the HDL-C level was higher than that before treatment. The full-term delivery rate, ovulation rate, and normal menstrual rate in the combined group were higher than those in the control group. After treatment, the LH level in the combined group was lower than that in the control group, and the FSH level was higher than that in the control group. After 1 month, 3 months, and 5 months of treatment, RI, PI, and ovarian volume were decreased, and the endometrial thickness was increased in both groups. Also, after 5 months of treatment, the RI, PI, and ovarian volume in the combined group were significantly lower than those in the control group, and the endometrial thickness was significantly higher than that in the control group. There was no statistically significant difference in the incidence of adverse reactions between the two groups.

The article "The Effects of Letrozole and Metformin Combined with Targeted Nursing Care on Ovarian Function, LH, and FSH in Infertile Patients with Polycystic Ovary Syndrome" was published in 2022. Journal: J Healthc Eng.

**Conclusion:**

The combination of letrozole and metformin with targeted nursing in the treatment of infertility patients with PCOS has better clinical effect and high safety. It can improve endometrial receptivity and ovarian reserve function and regulate LH and FSH levels.

## 1. Introduction

Polycystic ovary syndrome (PCOS) is a common gynecological endocrine disorder in women of gestational age and the most common cause of female infertility. PCOS is characterized by oligomenorrhea, disorders, amenorrhea, ovulatory dysfunction, infertility, and hyperandrogenism symptoms [1]. Due to the increasing pressure of women's life and work and the influence of living environment, the clinical incidence of PCOS is on the rise, which seriously affects the physical and mental health and life quality of patients [2]. The pathogenesis of PCOS is unclear but may be related to hyperandrogenemia, hyperinsulinemia, luteinizing hormone/follicle-stimulating hormone ratio imbalance, metabolic abnormalities, inflammation, advanced glycation end products, and endoplasmic reticulum stress [3–5]. PCOS is frequently associated with obesity, type 2 diabetes and gestational diabetes, cardiovascular disease, hepatic steatosis, and endometrial cancer [6–8]. These diseases pose a serious threat to women's lives.

At present, the clinical treatment of PCOS mainly includes menstrual cycle regulation, antihyperandrogenemia treatment, weight control, management of insulin resistance and metabolic disorders, and lifestyle changes [9, 10]. The drug used for clinical symptomatic treatment to reduce insulin resistance in PCOS patients is usually metformin [11]. Metformin can reduce the level of insulin resistance in patients, improve insulin sensitivity, reduce hepatic glucose production, and promote the normalization of glucose metabolism. In recent years, letrozole tablets have some applications in the treatment of PCOS and have the effect of ovulation induction [12]. However, there are few studies on the effects of letrozole tablets and metformin tablets on ovarian function in patients with polycystic ovary infertility. In the treatment of PCOS patients, it is important to take appropriate nursing measures for the patient while ensuring the efficacy of the drug. Targeted nursing [13] mainly provides systematic nursing measures for patients from the aspects of psychology, health, and sports. It provides more accurate targeted services for patients, improves patient prognosis, and increases the probability of later pregnancy. Therefore, this study aimed to investigate the effect of letrozole and metformin combined with targeted nursing on sex hormone levels and pregnancy rate in infertile patients with PCOS.

The article "The Effects of Letrozole and Metformin Combined with Targeted Nursing Care on Ovarian Function, LH, and FSH in Infertile Patients with Polycystic Ovary Syndrome" was published in 2022. Journal: J Healthc Eng.

## 2. Materials and Methods

### 2.1. Patients

A total of 72 patients with PCOS from April 2019 to February 2021 were collected. According to different treatment methods, they were divided into a combined group and a control group, with 36 cases in each group. The age of the combined group was 23 to 37 years old, with an average age of 29.81 ± 3.52 years old. The period of infertility was 1.0 to 3.5 years, with an average of 2.38 ± 0.61 years. The BMI was 24.20 ± 4.67 kg/m^2^. The age of the control group was 24–39 years old, with an average age of 30.78 ± 3.63 years. The infertility years ranged from 1.0 to 3.9 years, with an average of 2.54 ± 0.74 years. The BMI was 24.66 ± 4.70 kg/m^2^. There was no significant difference in age, years of infertility, and BMI between the two groups (*P* > 0.05).

### 2.2. Inclusion Criteria

1. The patient meets clinical criteria for polycystic ovary infertility [14].
2. Confirmation of the diagnosis of PCOS and infertility by combining the patient's clinical manifestations, signs, sex hormone detection, B-ultrasound, and other imaging examinations.
3. The patient meets the treatment indications of Trazole combined with metformin.
4. Patients have fertility requirements.
5. Patients and their families gave informed consent and signed an informed consent form.

### 2.3. Exclusion Criteria

1. The patient has other diseases of the female reproductive system such as tubal obstruction, stenosis, cervicitis, and uterine fibroids.
2. The patient has other diseases of reproductive or endocrine system.
3. The patient has chronic diseases such as liver, kidney, heart, and lung insufficiency.
4. Patients are allergic to the drugs used in this study.
5. Patients suffer from mental illness or poor compliance.

### 2.4. Treatment

The control group was given metformin hydrochloride tablets (national medicine Zhunzi H20023370, Sino-US Shanghai Squibb Pharmaceutical Co., Ltd., 0.5 g/time, 3 times/d). On the basis of the control group, letrozole tablets (Guoyao Zhunzi H19991001, Jiangsu Hengrui Medicine Co., Ltd., 2.5 mg/time, 1 time/d) were given orally in the combination group. It starts on the 5th day of menstruation and lasts for 5 days. Both groups were treated continuously for 5 menstrual cycles.

Both groups were given targeted nursing [15]. The specific method is as follows:

1. Preliminary diagnosis and examination: patients should be informed of the diagnosis and treatment process, such as cost, technical methods, and routine examinations. Various forms of education should be performed to improve patients' compliance with treatment and help patients build up their self-confidence.
2. Treatment: due to the complicated treatment plan of PCOS patients, nursing staff should strengthen the medication guidance for patients and patiently explain the usage and dosage of drugs, drug contraindications, common adverse reactions, and treatment methods. Nursing staff should make a self-made medication record form and inform the patient to fill it out after taking the medication every day so as to supervise the patient's medication status and lay the foundation for subsequent treatment.
3. Continuous nursing intervention: nursing staff should provide patients with effective nursing support in terms of diet, exercise, and psychology. First, a dietary plan should be developed based on the patient's age, weight, condition, and activity level to limit fat and sugar intake. Daily intake of fat should be 25% to 35% or less of total calories. Patients are encouraged to consume moderate amounts of protein and to eat more fresh, low-sugar fruits and vegetables. Second, patients are instructed to perform rhythmic aerobic exercise, such as cycling, aerobics, and brisk walking. Aerobic exercise time should be controlled between 30 and 60 minutes. Also, it should be no less than 3 times a week, and 5 to 7 times is ideal. Finally, nursing staff should understand the patient's psychological status, correct their misunderstandings, inform patients of the importance of a positive attitude, and encourage patients with successful cure cases.
4. Luteal support and failure support: if the pregnancy test fails after treatment, the nurse should arrange a return visit to give the patient psychological comfort. After a successful pregnancy test, the patient was told to use luteal support drugs. Also, patients were given dietary guidance.

The article "The Effects of Letrozole and Metformin Combined with Targeted Nursing Care on Ovarian Function, LH, and FSH in Infertile Patients with Polycystic Ovary Syndrome" was published in 2022. Journal: J Healthc Eng.

### 2.5. Clinical Efficacy

The effective rate of the treatment includes the sum of significant effect and remission.

Significantly effective: after treatment, the clinical symptoms of polycystic ovary were significantly improved, and the menstrual time returned to normal. Ovulation recovered well, and the cervix was in good condition. The patient can fertilize or even become pregnant normally, and there are no obvious complications or adverse reactions after treatment.

Remission: after treatment, the clinical symptoms caused by polycystic ovary were effectively controlled, and menstruation returned to normal. Ovulation function and cervical condition were effectively restored. Also, there were minor complications or adverse reactions but could be controlled after treatment.

Ineffective: the clinical symptoms caused by polycystic ovary in the patient did not improve significantly after treatment. Patients have irregular menstruation, less ovulation, and poor cervical condition. Patients cannot fertilize and conceive normally, or experience serious complications and adverse reactions.

### 2.6. Ovarian Endocrine Function Index

The ovarian endocrine function indexes, including luteinizing hormone (LH) and follicle-stimulating hormone (FSH), were compared between the two groups before treatment and after 5 menstrual cycles. LH and FSH were detected using an automatic biochemical analyzer (model: i-2000, Abbott Company, USA) in strict accordance with the product instructions. 3 mL of fasting venous blood was drawn and centrifuged at 3000 r/min for 5 min. LH and FSH were measured by the chemiluminescence immunoassay using related detection kits (Shanghai Yili Biotechnology Co., Ltd).

### 2.7. Glycolipid Metabolism Index

The glucose and lipid metabolism indexes of the two groups were compared before treatment and after 5 menstrual cycles of treatment. The changes of triglyceride (TG), total cholesterol (TC), and high-density lipoprotein cholesterol (HDL) levels were measured by using an automatic biochemical analyzer. The levels of glycosylated hemoglobin (HbA1c), fasting insulin (FINS), and insulin resistance index (HOMA-IR) were detected by the enzyme-linked immunosorbent assay (ELISA).

### 2.8. Color Doppler Ultrasound

Blood flow resistance index (RI), blood flow pulsatility index (PI), endometrial thickness, and ovarian volume were measured by transvaginal color Doppler ultrasound before treatment, 2 months, and 3 months after treatment.

### 2.9. Other Indices

The full-term delivery rate, ovulation rate, and normal menstrual rate after 5 menstrual cycles were compared between the two groups. The adverse reactions of the patients were observed and recorded, including nausea and vomiting, diarrhea, abnormal liver function, abnormal renal function, and headache.

### 2.10. Statistical Analysis

The SPSS 23.0 software was used for statistical analysis in this study. All experiments were performed in triplicate. The enumeration data were compared using *χ*2 test and expressed as frequency (*n* (%)). *P* < 0.05 was considered statistically significant.

## 3. Results

### 3.1. Comparison of Clinical Efficacy between the Two Groups

There were 34 effective cases in the combined group, and the total effective rate was 94.44%. There were 29 effective cases in the control group, and the total effective rate was 80.56%. The difference between the two groups was statistically significant (*P* < 0.05, Table 1).

### 3.2. Comparison of serum glucose and lipid metabolism in two groups of patients before and after treatment

As shown in Figure 1, the levels of HbA1c, FINS, and HOMA-IR in the two groups after treatment were lower than those before treatment (*P* < 0.05), and the reduction in the combined group was more significant (*P* < 0.05). As shown in Figure 2, the levels of TG and TC in the two groups after treatment were lower than those before treatment (*P* < 0.05), and the levels of HDL-C were higher than those before treatment (*P* < 0.05). After treatment, the levels of TG and TC in the combined group were lower than those in the control group, and the level of HDL-C was higher than that in the control group (*P* < 0.05, Figure 2).

The article "The Effects of Letrozole and Metformin Combined with Targeted Nursing Care on Ovarian Function, LH, and FSH in Infertile Patients with Polycystic Ovary Syndrome" was published in 2022. Journal: J Healthc Eng.

### 3.3. Comparison of pregnancy status, ovulation rate, and normal menstrual rate between two groups of patients

The full-term delivery rate, ovulation rate, and normal menstrual rate in the combined group were higher than those in the control group, and the differences were statistically significant (*P* < 0.05, Table 2).

### 3.4. Comparison of LH and FSH Levels before and after Treatment in the Two Groups

There was no significant difference in LH and FSH levels between the two groups before treatment (*P* > 0.05, Figure 3). After treatment, the LH level in the combined group was lower than that in the control group, and the FSH level was higher than that in the control group (*P* < 0.05, Figure 3).

### 3.5. Comparison of Endometrial Receptivity between the Two Groups before and after Treatment

There was no significant difference in RI, PI, endometrial thickness, and ovarian volume between the two groups before treatment (*P* > 0.05, Figure 4). At 1 month, 3 months, and 5 months after treatment, RI, PI, and ovarian volume were decreased, and endometrial thickness was increased in both groups. After 5 months of treatment, the RI, PI, and ovarian volume in the combined group were significantly lower than those in the control group, and the endometrial thickness was significantly higher than that in the control group (*P* < 0.05, Figure 4).

### 3.6. Comparison of Adverse Reactions in the Two Groups

The number of nausea and vomiting, and diarrhea in the combined group was 4 and 2, respectively. The number of nausea and vomiting, diarrhea, and headache in the control group was 3, 3, and 1, respectively. There was no significant difference in the incidence of adverse reactions between the two groups (*P* > 0.05, Table 3).

## 4. Discussion

PCOS is a common gynecological disease with endocrine disorders and metabolic dysfunction. With the increase of clinical incidence, PCOS has become an important cause of infertility in pregnant women, which seriously affects the health and safety of patients and family life [16]. It has been shown that infertility in PCOS patients is associated with high levels of luteinizing hormone, hypothalamic-pituitary-ovarian axis disorders, ovulation disorders, and hyperandrogenism [17]. Endometrial receptivity is the receptivity of the endometrium to the embryo, which is limited by time and space. During a normal reproductive cycle, the endometrium is the most receptive. When PCOS patients are in a state of infertility antagonism for a long time, a large number of androgen receptors will act on the patient's endometrium [18], thereby reducing the receptivity of the endometrium and leading to implantation failure.

The article "The Effects of Letrozole and Metformin Combined with Targeted Nursing Care on Ovarian Function, LH, and FSH in Infertile Patients with Polycystic Ovary Syndrome" was published in 2022. Journal: J Healthc Eng.

At present, the pathogenesis of PCOS remains unclear. It is generally believed that the occurrence of PCOS is related to factors such as hyperinsulinemia, adrenal endocrine disorders, hypothalamic-pituitary-ovarian axis regulation dysfunction, and endocrine dysfunction [19]. Metformin reduces insulin resistance by increasing insulin sensitivity in the liver and peripheral tissues. Metformin is currently the most widely used drug for the treatment of metabolic and endocrine disorders in PCOS [20], which improves ovarian steroid synthesis and reduces circulating androgen levels. For patients with polycystic ovary infertility, in addition to ovulation induction, the fundamental purpose of the treatment is to improve the pregnancy rate. Letrozole [21–23] is a new type of ovulation induction drug, belonging to the third generation nonsteroidal aromatase inhibitors. Inhibition of aromatase blocks the synthesis and conversion of androgens to estrogens, thereby rapidly regulating androgen and estrogen levels in PCOS patients. In addition, letrozole has been found to be effective in maintaining normal secretion of cervical mucus and creating a favorable environment for embryo implantation by promoting endometrial growth [24]. However, due to the long process of drug treatment, the patient's physiological and psychological states are prone to changes, which may have a great impact on the treatment effect. Routine nursing intervention is difficult to meet the needs of patients with physical and psychological service. Lack of targeted nursing measures is not conducive to the improvement of clinical efficacy. Targeted nursing [25] divides the treatment of PCOS patients into multiple stages, and the nursing measures are more comprehensive and targeted. Patients can clearly understand the details of their own treatment, which helps patients stabilize emotional changes and improve disease prognosis. Not only that, targeted nursing intervention starts from the needs of patients for medical services, and focuses on the nursing problems of patients' physical and mental aspects. Strengthening nursing intervention for patients during treatment can stabilize patients' emotions, improve their medical behavior, and help improve pregnancy outcomes.

The article "The Effects of Letrozole and Metformin Combined with Targeted Nursing Care on Ovarian Function, LH, and FSH in Infertile Patients with Polycystic Ovary Syndrome" was published in 2022. Journal: J Healthc Eng.

LH and FSH are indicators of sex hormones, and the combined action of LH and FSH can promote follicle maturation as well as the formation and maintenance of the corpus luteum [26, 27]. This study found that the changes of serum LH and FSH levels in the combined group after treatment were significantly higher than those in the control group, confirming that letrozole combined with metformin is more effective in the treatment of polycystic ovary infertility and can improve the LH and FSH levels of patients. The results of this study showed that letrozole combined with metformin can improve endometrial receptivity and promote physical recovery in patients. In addition, letrozole tablets can improve the success rate of ovulation induction, term delivery rate, and normal menstrual rate by regulating the negative feedback of the hypothalamic-pituitary axis. In this study, color Doppler ultrasonography was used to examine endometrial thickness, ovarian volume, RI, and PI in PCOS patients before and after treatment. Compared with the control group, the endometrial thickness in the combination group was increased, and the ovarian volume, RI, and PI were decreased after treatment, indicating that metformin combined with letrozole treatment can further improve the ovarian status of patients and treat infertility patients. PCOS is closely related to the disorder of glucose and lipid metabolism. The results of this study showed that after treatment, serum HbA1c, FINS, HOMA-IR, TG, and TC levels in the combined group were significantly lower than those in the control group, and HDL-C level was significantly higher than that in the control group. It is suggested that letrozole and metformin combined with targeted nursing in the treatment of PCOS can effectively improve the level of glucose and lipid metabolism in patients and improve the therapeutic effect. However, the sample size used in this study is relatively small. We will expand the sample size to further confirm our conclusions in the future.

## 5. Conclusion

To sum up, letrozole and metformin combined with targeted nursing can improve endometrial receptivity in infertile patients with PCOS, and more effectively improve ovarian dysfunction and glucose and lipid metabolism. Its effect is remarkable, and it is worth promoting and applying.

## Figures and Tables

**Figure 1:** Comparison of blood glucose levels between the two groups before and after treatment. (a) The comparison of HbAlc levels between the two groups before and after treatment (*n* = 36). (b) The comparison of FINS level between the two groups before and after treatment (*n* = 36). (c) The comparison of HOMA-IR levels between the two groups before and after treatment (*n* = 36) (^*∗*^*P* < 0.05).

The article "The Effects of Letrozole and Metformin Combined with Targeted Nursing Care on Ovarian Function, LH, and FSH in Infertile Patients with Polycystic Ovary Syndrome" was published in 2022. Journal: J Healthc Eng.

**Figure 2:** Comparison of blood lipid levels between the two groups before and after treatment. (a) The comparison of TG levels between the two groups before and after treatment (*n* = 36). (b) The comparison of TC levels between the two groups before and after treatment (*n* = 36). (c) The comparison of HDL-C levels between the two groups before and after treatment (*n* = 36) (^*∗*^*P* < 0.05).

**Figure 3:** Comparison of LH and FSH levels between the two groups before and after treatment. (a) The comparison of LH levels between the two groups before and after treatment (*n* = 36). (b) The comparison of FSH levels between the two groups before and after treatment (*n* = 36) (^*∗*^*P* < 0.05).

**Figure 4:** Comparison of endometrial receptivity between the two groups before and after treatment. (a) The RI comparison of the two groups at 1, 3, and 5 months before treatment (*n* = 36). (b) The PI comparison between the two groups at 1, 3, and 5 months before treatment (*n* = 36). (c) The comparison of endometrial thickness between the two groups at 1, 3, and 5 months before treatment (*n* = 36). (d) The comparison of ovarian volumes between the two groups at 1, 3, and 5 months before treatment (*n* = 36) (^*∗*^*P* < 0.05).

**Table 1:** Comparison of clinical efficacy between the two groups.

Group	*n*	Significantly effective	Remission	Ineffective	Total effective rate
Combined group	36	22	12	2	34 (94.44)
Control group	36	11	18	7	29 (80.56)
*X* ^2^					7.644
*P* value					<0.05^*∗*^

**Table 2:** Comparison of pregnancy status, ovulation rate, and normal menstrual rate between the two groups (*n* (%)).

Group	n	Pregnancy status	Ovulation rate	Normal menstrual rate
Combined group	36	31 (86.11)	32 (88.89)	33 (91.67)
Control group	36	23 (63.89)	25 (69.44)	26 (72.22)
*X* ^2^		4.741	4.126	4.600
*P* value		0.029^*∗*^	0.042^*∗*^	0.032^*∗*^

^*∗*^ *P* < 0.05.

**Table 3:** Comparison of adverse reactions in the two groups.

Group	*n*	Nausea and vomiting	Diarrhea	Abnormal liver function	Abnormal kidney function	Headache
Combined group	36	4	2	0	0	0
Control group	36	3	3	0	0	1

## Data Availability

The data used to support the findings of this study are available from the corresponding author upon request.

## References

[1] Azziz R. (2018). Polycystic ovary syndrome. *Obstetrics & Gynecology*.

[2] Meier R. K. (2018). Polycystic ovary syndrome. *Nursing Clinics of North America*.

The article "The Effects of Letrozole and Metformin Combined with Targeted Nursing Care on Ovarian Function, LH, and FSH in Infertile Patients with Polycystic Ovary Syndrome" was published in 2022. Journal: J Healthc Eng.

[3] Bednarska S., Siejka A. (2017). The pathogenesis and treatment of polycystic ovary syndrome: what’s new?. *Advances in Clinical and Experimental Medicine*.

[4] Ortiz-Flores A. E., Luque-Ramírez M., Escobar-Morreale H. F. (2019). Polycystic ovary syndrome in adult women. *Medicina Clínica*.

[5] Escobar-Morreale H. F. (2018). Polycystic ovary syndrome: definition, aetiology, diagnosis and treatment. *Nature Reviews Endocrinology*.

[6] Patel S. (2018). Polycystic ovary syndrome (PCOS), an inflammatory, systemic, lifestyle endocrinopathy. *The Journal of Steroid Biochemistry and Molecular Biology*.

[7] ACOG committee opinion (1998). Obstetrician-gynecologists’ ethical responsibilities, concerns, and risks pertaining to adoption. Number 194, November 1997. Committee on Ethics. American College of Obstetricians and Gynecologists. *International Journal of Gynaecology & Obstetrics*.

[8] Zhang J., Bao Y., Zhou X., Zheng L. (2019). Polycystic ovary syndrome and mitochondrial dysfunction. *Reproductive Biology and Endocrinology*.

[9] Jin P., Xie Y. (2018). Treatment strategies for women with polycystic ovary syndrome. *Gynecological Endocrinology*.

[10] Rocha A. L., Oliveira F. R., Azevedo R. C. (2019). Recent advances in the understanding and management of polycystic ovary syndrome. *F1000Research*.

[11] Morley L. C, Tang T, Yasmin E, Norman R. J, Balen A. H (2017). Insulin-sensitising drugs (metformin, rosiglitazone, pioglitazone, D-chiro-inositol) for women with polycystic ovary syndrome, oligo amenorrhoea and subfertility. *Cochrane Database of Systematic Reviews*.

[12] Amer S. A., Smith J., Mahran A., Fox P., Fakis A. (2017). Double-blind randomized controlled trial of letrozole versus clomiphene citrate in subfertile women with polycystic ovarian syndrome. *Human Reproduction*.

[13] Tay C. T., Pirotta S., Teede H. J. (2021). Polycystic ovary syndrome models of care: a review and qualitative evaluation of a guideline-recommended integrated care. *Seminars in Reproductive Medicine*.

[14] Belenkaia L. V., Lazareva L. M., Walker W., Lizneva D. V., Suturina L. V. (2019). Criteria, phenotypes and prevalence of polycystic ovary syndrome. *Minerva Ginecologica*.

[15] Tay C. T, Moran L. J, Wijeyaratne C. N (2018). Integrated model of care for polycystic ovary syndrome. *Seminars in Reproductive Medicine*.

[16] Rosenfield R. L. (2020). Current concepts of polycystic ovary syndrome pathogenesis. *Current Opinion in Pediatrics*.

[17] Osibogun O., Ogunmoroti O., Michos E. D. (2020). Polycystic ovary syndrome and cardiometabolic risk: opportunities for cardiovascular disease prevention. *Trends in Cardiovascular Medicine*.

The article "The Effects of Letrozole and Metformin Combined with Targeted Nursing Care on Ovarian Function, LH, and FSH in Infertile Patients with Polycystic Ovary Syndrome" was published in 2022. Journal: J Healthc Eng.

[18] Macut D., Bjekić-Macut J., Rahelić D., Doknić M. (2017). Insulin and the polycystic ovary syndrome. *Diabetes Research and Clinical Practice*.

[19] Otto-Buczkowska E., Grzyb K., Grzyb K., Jainta N. (2018). Polycystic ovary syndrome (PCOS) and the accompanying disorders of glucose homeostasis among girls at the time of puberty. *Pediatric Endocrinology, Diabetes and Metabolism*.

[20] Practice M. (2012). Committee of American society for reproductive, multiple gestation associated with infertility therapy: an American society for reproductive medicine practice committee opinion. *Fertility and Sterility*.

[21] Najafi P. Z., Noghabi S. P., Afzali N., Mohammadzadeh S. (2020). Comparing the effect of clomiphene citrate and letrozole on ovulation induction in infertile women with polycystic ovary syndrome. *JPMA. The Journal of the Pakistan Medical Association*.

[22] Franik S., Eltrop S. M, Kremer J. A., Kiesel L., Farquhar C. (2018). Aromatase inhibitors (letrozole) for subfertile women with polycystic ovary syndrome. *Cochrane Database of Systematic Reviews*.

[23] Mejia R. B., Summers K. M., Kresowik J. D., Van Voorhis B. J. (2019). A randomized controlled trial of combination letrozole and clomiphene citrate or letrozole alone for ovulation induction in women with polycystic ovary syndrome. *Fertility and Sterility*.

[24] Shi S., Hong T., Jiang F., Zhuang Y., Chen L., Huang X. (2020). Letrozole and human menopausal gonadotropin for ovulation induction in clomiphene resistance polycystic ovary syndrome patients. *Medicine (Baltimore)*.

[25] Torres-Zegarra C., Sundararajan D., Benson J. (2021). Care for adolescents with polycystic ovary syndrome: development and prescribing patterns of a multidisciplinary clinic. *Journal of Pediatric and Adolescent Gynecology*.

[26] Saadia Z. (2020). Follicle stimulating hormone (LH: FSH) ratio in polycystic ovary syndrome (PCOS) - obese vs. Non- obese women. *Medical Archives*.

[27] Laven J. S. E. (2019). Follicle stimulating hormone receptor (FSHR) polymorphisms and polycystic ovary syndrome (PCOS). *Frontiers in Endocrinology*.

